The article "The Effect of Biofeedback Therapy Combined with Comprehensive Nursing Intervention on the Quality of Life of Patients with Functional Constipation Based on Dynamic Magnetic Resonance Defecation" was published in 2021. Journal: J Healthc Eng.

# The Effect of Biofeedback Therapy Combined with Comprehensive Nursing Intervention on the Quality of Life of Patients with Functional Constipation Based on Dynamic Magnetic Resonance Defecation

**DOI:** 10.1155/2021/9947373

**Published:** 2021-05-13

**Authors:** Zhongshao Kuang, Shuangyuan Dai, Yinjuan Xiao, Weio Luo, Jing Tian, Ashutosh Sharma, Shailendra Tiwari, Manish Gupta, Manjit Kaur, Mohd Asif Shah

**Affiliations:** ^1^The Third Affiliated Hospital of South China University, Hengyang, Hunan 421999, China; ^2^Affiliated Hospital of Northwest Minzu University, Lanzhou, Gansu 730030, China; ^3^Institute of Computer Technology and Information Security, Southern Federal University, Rostov-on-Do, Russia; ^4^Thapar Institute of Engineering and Technology, Patiala, India; ^5^Computer Science and Engineering Department, Moradabad Institute of Technology, Moradabad, India; ^6^Computer Science Engineering, School of Engineering and Applied Sciences, Bennett University, Greater Noida 201310, India; ^7^Bakhtar University, Kabul, Afghanistan

## Abstract

In order to study the quality of life of patients with functional constipation based on dynamic magnetic resonance defecation, the biofeedback therapy combined with comprehensive nursing intervention was used to diagnose and treat the patients, so as to explore its clinical efficacy and its impact on patients' quality of life. The obstructed defecation surgical treatment carries frequent recurrences, and dynamic magnetic resonance imaging defecography evaluated and elucidated the underlying anatomic features. This research selected 80 patients who came to our hospital for treatment of functional constipation and evaluated and recorded various clinical indicators before and after treatment in the form of questionnaire survey. The results showed that the clinical symptom scores of patients with functional constipation before and after treatment were greatly different (*P* < 0.05). Thus, the biofeedback therapy combined with comprehensive nursing intervention showed a good clinical effect in the treatment of patients with functional constipation and significantly improved the quality of life of patients, showing high clinical application and promotion value. A convenient diagnostic procedure is represented by the dynamic magnetic resonance imaging in females, especially pelvic floor organs dynamic imaging during defecation.

## 1. Introduction

Functional constipation (FC) has become a very common chronic functional gastrointestinal disease in modern life [1]. Due to poor living habits and unhealthy diet, the incidence of the disease is increasing year by year, which has a serious impact on the body and psychology of the sick patients. According to research, the incidence of constipation over 18 years old in Beijing, Guangzhou, Tianjin, Nanchang, and other places is 6.07%, 4%, 11.6%, and 3.3%, respectively [2, 3]. This shows that constipation occurs in a wide range of groups, and people of any age group have a certain chance of getting sick. The specific clinical manifestations of FC include difficulty in defecation, inconstant defecation, and abdominal pain [4, 5]. According to the current level of diagnosis and treatment, there is no clinically specific medicine for the treatment of functional constipation. Generally, the commonly used treatment method is oral diarrhea medicine and external application of medicine, but these two treatment methods have not been particularly obvious [6, 7]. Now our hospital uses biofeedback (BF) therapy combined with nursing intervention to treat FC in order to find the most effective clinical treatment. MRI functional constipation is shown in Figure 1.

The article "The Effect of Biofeedback Therapy Combined with Comprehensive Nursing Intervention on the Quality of Life of Patients with Functional Constipation Based on Dynamic Magnetic Resonance Defecation" was published in 2021. Journal: J Healthc Eng.

BF is also called biofeedback training. The therapy uses a biofeedback mechanism to collect, process, and amplify the patient's own physiological activity information through the use of a biofeedback mechanism, adjusting physiological activities according to the observed information of their own physiological activities, so as to reduce or eliminate abnormal physiological changes. Therefore, it is an emerging biological behavior therapy method [8–10]. The use of BF in FC is actually the use of sound and image feedback to stimulate the brain to regulate the body, so as to achieve control and prevent the occurrence of constipation [11–14]. This therapy was proposed by Brik in 1973, and then Bleijenberg applied it to patients with chronic constipation [15, 16]. With continuous improvement and development, BF has gradually become a general treatment plan for treating FC patients.

The diagnosis also plays a great role in the treatment of FC patients [17]. The common way to diagnose patients with constipation is to observe whether the patient has pelvic floor dysfunction by dynamic magnetic resonance defecation [18, 19]. Dynamic magnetic resonance defecation technology has not appeared in China for a long time, but it has developed rapidly. The amount of information about the condition provided by it is relatively comprehensive, which provides an important basis for doctors to diagnose the cause of the condition of patients with constipation. In the evaluation of pelvic floor dysfunction, it has now become the best imaging examination method [20].

From the rectum, contents are evacuated and it is collectively described by the collective noun known as obstructed defecation (OD). In the Western world, OD prevalence is 7% in the adult population and it is more frequent in females. During the fourth and fifth decade of life, there is defecation difficulty and the OD pathophysiology is unknown [21]. Due to defective rectal filling and sensation, functional outlet obstruction, pelvic floor problem is difficult. The cornerstone of clinical evaluation of patients is represented by the physical examination and the detailed history. For diagnosis and treatment planning of outlet obstruction, different anorectal physiology testings are recommended which depends on the local situation and availability. The nonspecific and overlapping symptoms are presented by the variety of pelvic floor pathologies which are comprised by the three compartments. Symptoms are like pelvic fullness, pain, and problems defecating [22]. The concomitant pathology is masked by the symptoms in various compartments and many of the patients undergo surgical repair symptoms from the unmasked problems. Without imaging, the majority of patients can be treated, but the severe symptoms patients can benefit from additional technical diagnostic procedures such as cinedefecography, colpocystodefecography, or magnetic resonance (MR) defecography.

The article "The Effect of Biofeedback Therapy Combined with Comprehensive Nursing Intervention on the Quality of Life of Patients with Functional Constipation Based on Dynamic Magnetic Resonance Defecation" was published in 2021. Journal: J Healthc Eng.

Before MR defecography imaging, patients have to take 600 mL of water over 30 minutes and better distend the small bowel, and thereby visualization is improved. Additionally, 20 mL IV injection of gadopentetate dimeglumine was administered through a butterfly needle [23]. Finally, immediately before image acquisition, small rectal catheter is used for instillation of 240 mL of aqueous sonographic gel into the rectum.

### 1.1. MRI Feature Analysis

In consensus retrospectively, two radiologists of the abdomen evaluated the images at a PACS workstation. They reviewed the midsagittal dynamic images and presented it in cine loop mode. By utilizing the MRI grading system which is published previously, they are evaluated by each phase [24]. A grade for thickness and location of intussusceptions are added for the system modification. An assigned score was calculated to incorporate the scoring system. A total score for each phase is generated by this evaluation as given in Table 1.

Images are reviewed in sequence from the four phases in which they are independently acquired and scored. The proper analysis of images is done with regard to vaginal, bladder descent, rectal descent, and rectocele size. There is a positive movement in millimeters if it is above the pubococcygeal line and if it is below, then it will be negative. For determining bladder descent, bladder base was the landmark. The rectal descent is determined by the anorectal junction.

The article "The Effect of Biofeedback Therapy Combined with Comprehensive Nursing Intervention on the Quality of Life of Patients with Functional Constipation Based on Dynamic Magnetic Resonance Defecation" was published in 2021. Journal: J Healthc Eng.

### 1.2. Contribution

The main contribution of this paper is the treatment of functional constipation, and we evaluated and recorded various clinical indicators before and after treatment in the form of questionnaire survey.

- The comprehensive nursing intervention is combined with the biofeedback therapy for the good efficiency of patient's treatment.
- To improve the quality of patient's life to show the high clinical application and promotion value.
- To observe if the patient has pelvic floor dysfunction by dynamic magnetic resonance defecation.

The rest of the paper is organized as follows.  Section 2 provides an overview of the exhaustive literature survey followed by a methodology adopted in Section 3. A detailed discussion of obtained results is in Section 4. Finally, concluding remarks are provided in Section 5.

## 2. Related Work

The role of dynamic magnetic resonance imaging defecography is evaluated and the underlying anatomic and pathophysiologic effects are elucidated in this study for the failure minimization [25]. Forty consecutive constipated patients with OD symptoms went for perineal examination, proctoscopy, anorectal manometry, and Dynamic MRI defecography. The 23 patients are examined by the dynamic MRI of the pelvic floor. The pelvic floor disorders are combined with dynamic MRI defecography for diagnosis with 70% clinical results. It is concluded that the convenient diagnostic procedure is represented by the dynamic magnetic resonance imaging which is lesser in males than females. Dynamic magnetic resonance imaging had clinical impact in OD to the clinical assessment. The usefulness of the defecation phase is assessed in this paper during dynamic MR defecography [26]. Images from rest, maximal sphincter contraction and squeezing, maximal straining, and defecation were evaluated and scored independently with a modified grading system. The presence and degree of bladder, vaginal, rectal descent and size of rectocele, and intussusceptions are included in the features evaluation. Additional information is yielded by the defecation phase imaging on the degree of pelvic abnormalities. During pregnancy, the clinical presentation of achalasia is obscured by the diagnosis of new cases as symptoms and physiological changes [13]. In pregnancy, the achalasia management is challenging and, for every case, the treatment is individualized in which the mother and the fetus welfare are considered. A diagnostic and therapeutic challenge is represented by the achalasia suffering pregnant women. The current diagnostic and therapeutic options are reviewed, and to guide treatment of future cases, management algorithm is presented. By anorectal assessments, the phenotypic variability is characterized in constipated patients. Assessment of rectal balloon expulsion, rectal sensation, and pelvic floor structure is done in 52 constipated women and 41 age-matched asymptomatic women [27]. After body mass index correction, 71% of variance is explained by the 3 principal components between the patients. A heterogeneous entity is comprised by the functional defecation disorders as demonstrated by the obtained observations. The MR defecography in anorectal dysfunction diagnostic accuracy is assessed in this work. The 30 patients are included for the MR defecography with ARD for MR defecography detection [28]. Detection of increased perineal is done in 70% cases and this technique is an essential diagnostic tool for the optimum management of anorectal dysfunction patients.

The article "The Effect of Biofeedback Therapy Combined with Comprehensive Nursing Intervention on the Quality of Life of Patients with Functional Constipation Based on Dynamic Magnetic Resonance Defecation" was published in 2021. Journal: J Healthc Eng.

## 3. Materials and Methods

The 80 patients who were diagnosed and treated for FC in Indira Gandhi Medical College and Hospital from September 2019 to September 2020 were selected as the research objects, including 52 male patients and 28 female patients.

### 3.1. Basic Data

Patients who voluntarily withdrew and transferred to another hospital were excluded. The BF comprehensive nursing intervention was adopted to treat patients and follow-up patients' postoperative effects and quality of life.

The inclusion criteria were defined as follows: patients aging 18∼70 years old; patients satisfying the Roman diagnostic criteria of BF; patients receiving more than 4 BF treatments; patients with complete clinical data and information before and after treatment; patients without history of mental illness; and patients with stable emotion.

The exclusion criteria were determined as follows: patients who withdrew and transferred for treatment due to personal reasons; patients with other serious diseases or infectious diseases; and patients who were eventually lost to follow-up after the BF treatment.

### 3.2. Research Methods

All 80 patients under investigation were examined by dynamic magnetic resonance defecation (DMRD) during the diagnosis process, and the results were confirmed to be FC patients by the MyoTrac SA9800 myoelectric biofeedback training therapy device [29].

#### 3.2.1. Biofeedback Therapy

DMRD image of a FC patient is shown in Figure 2. Before BF treatment, the patient needs to understand the mechanism of human body function. Let the patient understand the mechanism of defecation and explain the anatomical characteristics of the anorectum, etc., and allow the patient to adjust to the state of excessive defecation. The digital anorectal examination was performed on the patient to know the dilation and contraction of the patient's anal sphincter. The training method adopts the side lying method, inserting the anal canal motor and a bile duct pressure measuring catheter into the anal canal and rectum, so that the patient's anorectal information could be displayed to the patient through a calculator [30]. At this time, the doctor's explanation and introduction allows the patient to distinguish the normal and abnormal images of the disease and finally guides the patient to learn and master the essentials of increasing intra-abdominal pressure and systolic pressure and relaxing the anus and repeat training in this way. The treatment is 3 times a week, each time is about 1 hour, and each course is 8 times. During treatment, patients are also required to conduct autonomous training at home.

The article "The Effect of Biofeedback Therapy Combined with Comprehensive Nursing Intervention on the Quality of Life of Patients with Functional Constipation Based on Dynamic Magnetic Resonance Defecation" was published in 2021. Journal: J Healthc Eng.

#### 3.2.2. Comprehensive Nursing Intervention

Comprehensive nursing intervention was to enable patients to better understand the condition and treatment methods. Through this all-round physical and mental care, patients can receive the treatment of constipation physically and psychologically. Comprehensive nursing intervention requires medical staff to clearly explain the specific operating procedures of BF and related principles of action to patients, to guide FC patients correctly by observing and telling patients' feelings and acceptance during the process and to guide their daily living habits and changing diet structure and exercise method. In terms of diet structure, doctors need to inform patients to change their original unreasonable diet and regularly remind patients to drink more water and eat as much fruits and vegetables as possible for food intake; at the psychological level, medical staff communicate through daily illnesses and establish a good relationship of trust with patients, discover patients' negative emotions in time, help patients solve problems, and enhance their confidence in disease cure. In health education, actively popularize relevant knowledge, treatment processes, and curative effects to patients, so that patients can increase their disease. To reduce the patient's sense of insecurity, biofeedback training needs to clearly explain the precautions of the treatment method to the patient to avoid the poor treatment effect caused by the inappropriate method in the treatment of constipation. After each course of treatment, the patient's condition should be followed up in time [31].

### 3.3. Patients and Methods

With the obstructed defecation syndrome, 30 patients are included in the current study (21 females and 9 males). The constipation management algorithm is followed by all the patients and the preoperative clinical evaluation is done. The Agachan constipation scoring system and modified obstructed defecation syndrome score (ODS-S) were used for the assessment of the patients. A gynecologic evaluation was performed in all the women. There is an exclusion of intestinal inertia with the anorectal surgery patients. All the patients give the written consent and are subjected to proctoscopy and rectosigmoidoscopy for the diagnosis of contributing abnormality and tumor. The assessment of colonic motility is subjected by all the patients during the period when 106 patients were seen with chronic idiopathic constipation. The squeeze anal canal pressures are determined by the Anorectal Manometry with a perfused eight-channel manometry Smartlab. The rectal balloon of Schuster probe patients is used to measure the three elements of rectal sensation. Algorithm of constipation and obstructed defecation management is shown in Figure 3.

The article "The Effect of Biofeedback Therapy Combined with Comprehensive Nursing Intervention on the Quality of Life of Patients with Functional Constipation Based on Dynamic Magnetic Resonance Defecation" was published in 2021. Journal: J Healthc Eng.

### 3.4. Dynamic Magnetic Resonance Imaging Defecography

By using a body-array-surface coil, Phillips Gyroscan system is used to perform MRI. A sitting position simulation is done to flex the patient's knees. The static and dynamic (functional) pulse sequences are combined and then three-plane scout images were obtained for pubic symphysis identification. By T2-weighted turbo spin-echo sequence, axial and sagittal slices are obtained. The sagittal, axial, and coronal planes images are obtained and analysis is done. After administration of gel enema into the rectum, there is a repetition of static and dynamic sequences. By widening of the anorectal angle and perineal descent, rectal evacuation was generally associated with pelvic floor relaxation as shown in Figure 4.

All younger than 45 years of age, during rectal evacuation, the puborectalis indentation on the posterior rectal wall was more rather than less pronounced. There is a reduction in patient's anorectal angle average change during evacuation and squeezing. Perineal descent is normal in 44%, reduced in 35%, and increased in 21% of patients.

### 3.5. Statistical Methods

The data processing of this study was analyzed by SPSS 19.0 version statistical software, the measurement data were expressed by the mean ± standard deviation (*x* ± *s*), and the count data were expressed by the percentage (%). Pairwise comparison uses analysis of variance. *P* < 0.05 indicates that the difference is statistically significant.

## 4. Results and Discussion

All the 102 patients meeting the criteria were finally included, and 80 patients completed the survey.

### 4.1. Basic Data of Patients

Among them, 52 were male patients (66.44%) and 28 were female patients (35.53%) as shown in Figure 5. The age range of the patients was 18∼70 years old; the average age of men was 47.45 ± 20.19, and the average age of women was 46.16 ± 17.34; the average weight of men and women was 76.55 ± 10.19 and 61.41 ± 10.78, respectively; the average height of men and women was 176.12 ± 10.56 and 159.72 ± 10.28, respectively, as shown in Figure 6 below. The patient's illness time was 15.58 ± 5.72, and the biofeedback treatment period was 15.9 ± 8.97, and the follow-up time was 2 ± 1.94 years as given in Figure 7.

The article "The Effect of Biofeedback Therapy Combined with Comprehensive Nursing Intervention on the Quality of Life of Patients with Functional Constipation Based on Dynamic Magnetic Resonance Defecation" was published in 2021. Journal: J Healthc Eng.

### 4.2. Evaluation of Clinical Symptoms of Two Groups of Patients before and after Treatment

It can be seen from Figure 8 that the follow-up of 80 patients before and after treatment showed that the patient's defecation interval before treatment was 3.79 ± 2.17 days, and the defecation interval after biofeedback treatment was 1.01 ± 0.73 days; the score of defecation dysfunction before and after treatment was 2.73 ± 2.01 and 0.53 ± 0.09, respectively; the patient's incomplete defecation before treatment was 4.81 ± 2.07, and the score after treatment was 0.99 ± 0.47. It can be seen that the scores of each symptom of the patients were obviously different from the scores before treatment with statistical difference (*P* < 0.05).

### 4.3. Evaluation of Clinical Efficacy for Two Groups of Patients

Figure 9 shows the results of the follow-up of patients after treatment. The results show that during the follow-up, 31 people thought the efficacy was good, 30 people thought it was effective, and 19 people thought it was ineffective; the total effective rate was 76%, and the total satisfaction was 57.43%. After BF treatment, 66 people had significant effects, 13 were effective, and 1 was ineffective. The total effective rate was 99%, and the total satisfaction rate was 97.88%.

### 4.4. Evaluation on Quality of Life of Patients

Figures 10 and 11 show the comparison of the quality of life of patients before and after treatment with BF. The specific indicators set are physiological function, physical function, physical pain, vitality, emotional function, mental health, social function, general health, and other indicators for feedback. Among them, the physical function, physical pain, emotional function, mental health, social function, and general health level of the patients were observably different from the results before treatment (*P* < 0.05). It shows that the quality of life of patients is greatly improved after BF treatment.

Due to the various causes of patients with FC and the long course of the disease, the current treatment methods cannot effectively treat the FC in the long term. However, BF has been more and more applied in the clinical treatment. BF is safe, has no side effects, and does not cause surgical trauma. It is playing an increasingly important role in the treatment of FC. Related studies have shown that BF training can improve the clinical symptoms of patients with constipation dramatically and also help to improve the physiological functions of the gastrointestinal tract in the patient's body and reduce the patient's anxiety. Because FC patients have been ill for a long time, the efficacy of BF has also been widely concerned by patients. The results of 80 FC patients in this study showed that within 2 years of BF treatment, the clinical symptoms and mental health of the patients have changed significantly, with a total effective rate of 99% and a satisfaction rate of 97.88%, which has a good effect.

The article "The Effect of Biofeedback Therapy Combined with Comprehensive Nursing Intervention on the Quality of Life of Patients with Functional Constipation Based on Dynamic Magnetic Resonance Defecation" was published in 2021. Journal: J Healthc Eng.

Studies have shown that the physiological functions of the digestive tract are affected by both the endocrine system and the autonomic nervous system, so mental factors are also particularly important in the treatment of patients with FC [32]. Comprehensive nursing intervention plays a supporting role here. By assessing the patient's mental state and mental health level, medical staff can give patients different nursing interventions, which can greatly improve the success rate of BF treatment. Nursing intervention can effectively reduce the patient's stress response, improve the patient's psychosocial state, and improve the patient's behavior in compliance with doctor's advice. Therefore, nursing workers should communicate and follow-up in time before and after BF, supervise and remind patients, regularly assess the clinical symptoms and psychological level of patients, and solve problems for patients in time, so as to improve the long-term efficacy of the treatment.

### 4.5. Comparison of Radiological Diagnosis with the Clinical Diagnosis

In 66.67% of males and 74.19% of females, there is a consistency of the radiological diagnosis with the clinical diagnosis. With the dynamic MRI, there is a significant difference over clinical diagnosis in the rectocele, ARA descent, intussusception, cystocele, and enterocele diagnosis as shown in Table 2.

The significant diagnostic value is shown by the dynamic MRI in the female population as compared to males. 90% of patients are multifactorial as obstructed defecation and have more than one finding; 3 findings are obtained by the 40% of patients and 4 findings are obtained by the 20% patients. The graphical representation is shown in Figure 12 for better visualization and analysis.

It is clear from Figure 13 that the radiological diagnostic values are 27.50%, 64.29%, 46.51%, 40.58%, and 100% better than the clinical diagnostic values for rectocele, cystocele, intussusceptions, ARA descent, and enterocele, respectively.

The article "The Effect of Biofeedback Therapy Combined with Comprehensive Nursing Intervention on the Quality of Life of Patients with Functional Constipation Based on Dynamic Magnetic Resonance Defecation" was published in 2021. Journal: J Healthc Eng.

## 5. Conclusion

In this study, 80 FC patients were selected. After the diagnosis of dynamic magnetic resonance defecography, BF comprehensive nursing intervention was used. Before and after treatment, the clinical symptoms and mental health of the patients were analyzed and compared, and the changes in the quality of life of the patients before and after treatment were evaluated further. The results showed that the clinical symptom scores of FC patients before and after treatment were much different (*P* < 0.05). The overall effective rate of BF is 99%, and the patient's overall satisfaction with the quality of life after treatment is 97.88%. It can be seen that in the treatment of FC patients, the BF comprehensive nursing intervention method has a good clinical effect, improves the quality of life of the patients, and has high clinical application and promotion value. The disadvantage of this research topic is that the selected patient sample size is small and there is a certain deviation. The scope of application of the research results is also relatively small. In subsequent studies, the sample size of patients will be increased and the scope of the study will be expanded to further explore the clinical application value of BF. In summary, the results of this article provide reference for the treatment of FC patients to a certain extent.

## Figures and Tables

**Figure 1:** MRI functional constipation.

**Figure 2:** DMRD image of a FC patient (female, 68 years old).

**Figure 3:** Algorithm of constipation and obstructed defecation management.

**Figure 4:** Pelvic floor relaxation.

**Figure 5:** Proportion of male and female patients.

**Figure 6:** Comparison of basic data of patients.

**Figure 7:** Medial data of patients.

**Figure 8:** Clinical symptoms of two groups of patients before and after treatment. Note: ^*∗*^ indicated the difference was observable in contrast to the score before treatment (*P* < 0.05). Note: A: defecation interval; B: fecal traits; C: difficulty defecation; D: incomplete defecation; E: anus and rectum obstruction.

**Figure 9:** Evaluation of clinical efficiency for two groups of patients.

**Figure 10:** Evaluation on quality of life of patients. Note: ^*∗*^ indicated there was an observable difference in contrast to the status before treatment (*P* < 0.05). Note: A, B, C, and D referred to physiological function, physical function, physical pain, and vitality, respectively.

**Figure 11:** Evaluation on quality of life of patients. Note: ^*∗*^ indicated there was an observable difference in contrast to the status before treatment (*P* < 0.05). Note: A, B, C, and D referred to the emotional function, mental health, social function, and general health, respectively.

The article "The Effect of Biofeedback Therapy Combined with Comprehensive Nursing Intervention on the Quality of Life of Patients with Functional Constipation Based on Dynamic Magnetic Resonance Defecation" was published in 2021. Journal: J Healthc Eng.

**Figure 12:** Clinical diagnosis and dynamic MRI diagnosis in patients with obstructed defecation patients. The improvement percentage of the radiological diagnostic values is calculated over clinical diagnostic values for rectocele, cystocele, intussusceptions, ARA descent, and enterocele as presented in Figure 13.

**Figure 13:** Percentage of improvement of the radiological diagnostic values.

**Table 1:** Grading and scoring of MRI findings.

Abnormality	Small		Moderate		Large	
	Characteristics or size (cm)	Score	Characteristics or size (cm)	Score	Characteristics or size (cm)	Score
Rectal descent	<3 (below pubococcygeal line)	0	3–6 (below pubococcygeal line)	1	>6 (below pubococcygeal line)	2
Vaginal descent	<3 (below pubococcygeal line)	1	3–6 (below pubococcygeal line)	2	>6 (below pubococcygeal line)	3
Bladder descent	<3 (below pubococcygeal line)	1	3–6 (below pubococcygeal line)	2	>6 (below pubococcygeal line)	3
Rectocele size	<2	1	2–4	2	>4	3

**Table 2:** Comparison between clinical diagnosis and dynamic MRI diagnosis in patients with obstructed defecation patients.

	Radiological		Clinical	
	No.	%	No.	%
Rectocele	30	80	3	58
Cystocele	11	28	6	10
Intussusception	16	43	9	23
ARA descent	28	69	15	41
Enterocele	5	14	0	0

## Data Availability

All the data are shared in the main manuscript.
